RETRACTED

# Intelligent Sports Video Classification Based on Deep Neural Network (DNN) Algorithm and Transfer Learning

**DOI:** 10.1155/2021/1825273

**Published:** 2021-11-24

**Authors:** Xiaoping Guo

**Affiliations:** Shaanxi Normal University, Xi'an, Shaanxi 710000, China

## Abstract

Traditional text annotation-based video retrieval is done by manually labeling videos with text, which is inefficient and highly subjective and generally cannot accurately describe the meaning of videos. Traditional content-based video retrieval uses convolutional neural networks to extract the underlying feature information of images to build indexes and achieves similarity retrieval of video feature vectors according to certain similarity measure algorithms. In this paper, by studying the characteristics of sports videos, we propose the histogram difference method based on using transfer learning and the four-step method based on block matching for mutation detection and fading detection of video shots, respectively. By adaptive thresholding, regions with large frame difference changes are marked as candidate regions for shots, and then the shot boundaries are determined by mutation detection algorithm. Combined with the characteristics of sports video, this paper proposes a key frame extraction method based on clustering and optical flow analysis, and experimental comparison with the traditional clustering method. In addition, this paper proposes a key frame extraction algorithm based on clustering and optical flow analysis for key frame extraction of sports video. The algorithm effectively removes the redundant frames, and the extracted key frames are more representative. Through extensive experiments, the keyword fuzzy finding algorithm based on improved deep neural network and ontology semantic expansion proposed in this paper shows a more desirable retrieval performance, and it is feasible to use this method for video underlying feature extraction, annotation, and keyword finding, and one of the outstanding features of the algorithm is that it can quickly and effectively retrieve the desired video in a large number of Internet video resources, reducing the false detection rate and leakage rate while improving the fidelity, which basically meets people's daily needs.

## 1. Introduction

With the continuous improvement of information technology, people's demand for video information resources has also increased, and how to do a good job of processing data and information has become one of the very important research topics of relevant units [1]. In the current stage of data analysis information, machine learning algorithms play an increasingly important role, and deep learning has become one of the hottest information processing technologies nowadays [2]. Deep learning is essentially a new technology evolved from traditional neural networks, is also a neural network model applied to prediction and classification, and can be applied to many different analysis scenarios. Compared with traditional neural networks, deep neural networks have stronger classification performance and simpler model training, especially in the context of improving server performance and increasing data processing, and deep neural networks have been widely used in audio, video, text, and image fields [3]. Neural network as a machine learning model is inspired by the concept of neuron in biology and is able to simulate neurons in the brain [4].

RETRACTED

The corresponding output is obtained by activation function or specific weights, and the obtained computational structure is input to the next neuron [5]. The reason for the slow development of neural networks in the previous period is that (1) neural network training requires a large amount of data, and in the past, when the amount of information data was small, the trained network was likely to have overfitting problems. In the context of the improvement of China's information construction level and the expanding application of information technology, the era of big data has arrived, and there is a large amount of data that can be applied to the training of neural networks [6]. (2) Before the neural network was widely used, there were many difficulties in training, and many trainings could not be completed, because the gradient divergence problem could not be solved, and this kind of problem has been solved effectively now, which has greatly improved the learning ability of deep neural network [7]. Before deep learning was applied to video processing on a large scale, it had already achieved great success in the field of image recognition, and the classification model based on convolutional neural networks can significantly improve the recognition accuracy of Image Net images compared with the traditional model [8].

On this basis, the application value of deep neural networks has begun to receive general attention from experts and scholars, such as gradual application in video, audio, and text [9]. For example, in text processing, recurrent neural networks have been widely used, because they embody good application advantages in processing temporal recursive information. The classification of single frames of video by convolutional neural networks has led to a significant improvement in video classification. And now, convolutional neural networks have been able to perform multiframe processing, and the combination of recurrent neural networks with convolutional neural networks will make the video processing performance of related algorithms even more powerful [10]. Previous research work usually builds video classification algorithms based on image classification algorithms, which usually treats each frame of a video as an image, extracts the features of the video frame, and obtains a fixed-length vector of real numbers with the help of bag-of-words model, and the related training work is handled by support vector machines, which can be trained by support vector machines to classify other video frames [11]. The algorithm model is trained by the support vector machine to classify other video frames [12]. After convolutional neural networks were widely used in image classification, support vector machines were replaced by convolutional neural networks, resulting in a classification algorithm for a single video frame. However, this algorithm cannot take into account the correlation between frames and cannot be separated from the essence of image classification technology [13]. In order to make full use of the correlation between frames, a study has established a three-dimensional convolutional layer, which consists of a convolutional processing of several consecutive frames; i.e., the input of several consecutive frames or a video can also achieve video classification and, based on the relationship between frames, can also improve the accuracy of video classification, further increasing the performance of video classification and retrieval [14]. Studies have shown that the computational overhead of the network is positively correlated with the number of parameters, so the optimization of the network parameter size is essential to improve the network performance.

RETRACTED

This study further extends the network structure of video classification and investigates the image classification retrieval model based on the Tensor Flow framework, which demonstrates high retrieval accuracy and classification accuracy in the image classification process and further simplifies the structure of the whole model. The fidelity refers to the degree of similarity between the extracted key frames and the corresponding video; i.e., the higher the fidelity is, the better the key frames are restored to the original video. Assuming that the shot S contains *n* frames, the key frame extraction algorithm extracts *m* key frames from them, which is denoted as *K* = {*f*1, *f*2, ...*fn*}, and compares them one by one with the shot *n* frames starting from the first key frame and takes the smallest value as the key frame reference value. In this paper, the shortcomings of existing methods are comprehensively analyzed in video retrieval, and corresponding improvement methods are proposed in shot segmentation, key frame extraction, video annotation methods, and query expansion methods. Combined with the characteristics of sports video, this paper proposes a key frame extraction method based on clustering and optical flow analysis, and experimental comparison with the traditional clustering method. The quality of video content description depends on the good or bad features, and people can use good features of the relevant use of video research in many aspects, such as video retrieval and video classification and a series of operations; not only that, the technology largely promotes the future development and practical application of video and video feature extraction to alleviate the direct impression on video analysis and application; that is, the basis and focus of video processing technology are about the feature extraction of video, and accurate feature recognition is the prerequisite for the annotation of video.

RETRACTED

### 1.1. Related Work

In recent years, with the continuous development of science and technology, content-based video retrieval has developed rapidly, and the main purpose of this retrieval is to search for similar videos in the video library based on the video related content provided by the user as the search condition [15]. In the work of content-based video retrieval, the main study is the extraction of video features using deep neural networks, the basis for processing and analysis of video is the extraction of video features, and the merit of the extracted features has a direct impact on the relevant description of video content, which has an important value for the application of video retrieval [16]. With the recent advances in hardware such as massively parallel computing multicore GPUs commonly used in general purpose computing, researchers are generally paying attention to neural networks.

The researchers classified more than 1 million high-resolution images from the database through a convolutional neural network, and the researchers found that using a convolutional kernel size of about 3 × 3 for image feature extraction in the CNN can achieve significant results. The researchers built the spatiotemporal network by utilizing two CNN structures, a spatial network using a single frame of images from the video for network input and a temporal network using multiple frames of optical streams for network input [17]. In other words, the spatial and temporal features of the video are extracted separately and merged into one at the end, and the features extracted in this way are used to classify and organize the video with remarkable results. From the current point of view, video feature extraction still relies on techniques related to image processing [18]. Image is a way to describe an objective object, which is a relatively common human information carrier, from which some information of the described object can be known. Generally speaking, people mainly describe images in terms of texture, color, and shape and other related features. For the extraction of texture features, there are two main forms of structure-based and statistics-based methods [19].

RETRACTED

In addition, the accuracy of feature extraction can be improved by using the transfer learning method. Among the abovementioned feature extraction, color features are not sensitive enough to perceive changes such as orientation of the image to capture local features of the target in the image. Texture is only a surface feature extraction method that does not fully reflect the properties of the object; therefore, it jointly proposed features that fuse texture and color features. In video feature extraction, the appropriate selection of key frames is a key aspect, and treating key frame features as video features based only on the image level will result in the loss of time-domain information of the video, so some people process the video directly to extract features [20]. A relatively advanced extraction technique for video features is proposed by a researcher, who proposes to extract video features through an improved dense trajectory. First, the video is densely sampled, and the feature points obtained in the frames are used for feature point tracking using optical flow, so that the corresponding features can be obtained along the trajectory. Although the accuracy of this approach is relatively high from the current point of view, it cannot be applied to the occasions with relatively high requirements of time response because of its complex algorithm, which cannot improve the time performance well.

When performing video retrieval, the underlying feature extraction of the video is commonly in the form of color features described in the previous section, represented as a color histogram. The color histogram approach is used to form the color histogram features of the video by integrating all pixel points within the same pixel region of the video during feature extraction. Although this method of extracting color histogram features can perform efficient video feature extraction in a short time, this method ignores information related to video features such as video texture and shape when extracting video features, resulting in large errors when using the extracted features for similarity matching [21]. At the same time, when using color histogram for video feature extraction, it is not sensitive enough to reflect the change of color in the video. If there are two essentially unrelated scenes in the video, but because the color features appearing in the two video scenes are more similar, when using the color histogram to extract the video color features, it will result in the color histogram extracted from the two scenes being extremely similar, thus causing errors in video retrieval.

RETRACTED

## 2. A Deep Neural Network Query Method Based on Ontology Semantic Expansion

### 2.1. Deep Neural Network Model

In this paper, an end-to-end design idea is adopted for the classification and retrieval of sports videos; i.e., the input is the data of the whole picture and the category of the output picture, and the whole classification process is done automatically by the system without human operations such as parameter setting. Deep neural Inception V3 is used as the base network, and the network parameters and network structure are slightly modified based on the characteristics of sports videos, and the modified network converges faster, and the accuracy of classification is improved. In neural networks, such a core problem becomes the reduction of the number of connection weights to reduce the complexity of the model; a very common method is to add a penalty term after the loss function, in order to reduce the complexity of the model, usually using a 2-parameter number, but the 2-parameter error makes the weights and thresholds sparse, and then usually use a 1-parameter number to penalize the weights and thresholds. This algorithm is an improvement of the penalty term algorithm. The algorithm is a Hessian matrix-based network pruning algorithm that first constructs a local model of the error surface and analyzes the impact of perturbations in the weights. By performing Taylor expansion on the error function,

(1) $$\begin{array}{c} \partial E={\left(\frac{\partial E}{\partial w}\right)}^{T}+\frac{1}{2}{\left(\partial H\right)}^{\left(1/2\right)}, \end{array}$$

where *H* is the Hessian matrix, *T* denotes the transpose of the matrix, *w* is the parameter in the neural network, and *E* is the training set error. A local minimum is obtained by an optimization algorithm (e.g., L-M algorithm), and then the first term of the above equation is 0. Neglecting the third higher-order infinitesimal term yields

(2) $$\begin{array}{c} \partial E=\frac{1}{2}{\left(\frac{\partial H}{\partial w}\right)}^{\left(1/2\right)}. \end{array}$$

This method can be written by setting one of the weights to 0; thus,

(3) $$\begin{array}{c} \frac{1}{2}{\left(\frac{\partial H}{\partial w}\right)}^{\left(1/2\right)}+\;{\left(\frac{\partial E}{\partial w}\right)}^{T}=0, \end{array}$$

eq is the unit vector, and only if the qth term is 1, the other terms are 0. When one of the weights or thresholds is set to 0, so that Δ*E* is minimized, we can obtain

(4) $$\begin{array}{c} \min{\left(\frac{1}{2}\frac{\partial H}{\partial w}\right)}^{\left(1/2\right)}+\partial w=0. \end{array}$$

*H* is the Lagrangian multiplier, and by taking the partial derivative of the function *L*, we can obtain Δ*w*, Δ*w* leading to the error as

(5) $$\begin{array}{c} L_{p}=\left(\frac{1}{2}-\frac{1}{w}\right){\left[H^{-1}\right]}_{qq}. \end{array}$$

According to the pruning algorithm, the 10 Inception modules of the deep neural network were trained. According to the introduction of the Inception v3 model above, the team added a bilinear structure to the Inception v3 model to reduce the dimensionality of the feature map. It is also found that the reduction of parameters accelerates the convergence speed. Therefore, for each inception module, two bilinear structures are removed in the experiments in this paper. In addition, it is found that the first few convolutional layers extract the low-dimensional features of the image, while the later convolutional layers extract the high-dimensional features, so the last convolutional layer of the original network is removed, and the high convolutional kernel channels of the first two convolutional layers and the low convolutional kernel channels of the last two convolutional layers are cut off, and the softmax layer of the original network is replaced by a Sigmoid fully connected layer. The structure and parameters of the redesigned network are shown in Figure 1. Experiments show that the modified network shows good performance in processing sports videos. For the classification results, the results with the model prediction probability over 0.75 are extracted as the annotated words of the current image frame, and for each video to be detected, the annotated words of all key frames are pooled, and the duplicate words are removed as the annotated word set of the video for subsequent retrieval operations.

RETRACTED

### 2.2. Keyword Fuzzy Query Based on Transfer Learning

Traditional information retrieval is based on ordinary sets and Boolean logic, and the information to be retrieved is expressed in the form of Boolean expressions for logical comparison with user input; such a retrieval method is logically simple and easy to implement; however, the keywords input by users is often natural languages with strong ambiguity, and the traditional retrieval model does not have the concept of relevance, and only when the content to be retrieved matches exactly the query words can it be successfully retrieved, as shown in Figure 2. For the retrieval system to perform accurate analysis, it must have natural language understanding capability.

Some current retrieval models inevitably cause semantic loss when dealing with natural language, and the retrieval results are mostly unsatisfactory. Ontologies, as a knowledge modeling tool, offer the possibility to improve retrieval systems. A video retrieval system is a retrieval system for users, and the ultimate goal is to ensure that users can retrieve the video information of interest. However, often the search terms users input into the retrieval system do not express what they want to express well, which requires the retrieval system to understand the user's intention “intelligently” and improve the hit rate of retrieval, which requires the use of query expansion techniques. Several query expansion methods are described below.

The transfer learning analysis starts with correlation analysis of words and phrases in all documents, calculating the relevance of each word or phrase pair based on cooccurrence, and when the user enters a keyword to search, the word with the highest relevance to the word to be searched is found among these related words and added to the set of query words for joint search. Word clustering is the clustering analysis of words based on their cooccurrences, which is used to expand the query. If two words are related to each other, then the chance of cooccurrence of these two words in the set is high. However, words often have multiple meanings, and for words with multiple meanings, clustering algorithms usually assign them to different clusters based on different word meanings, resulting in less accurate query results and affecting the accuracy of retrieval.

Indexing potential semantic indexing is assuming that words in high-dimensional space can be represented using low-dimensional space. This technique uses singular value decomposition (SVD) method, which is a dimensionality reduction technique. Assume that, given a word frequency matrix *M* × *N* of *M* words and *N* documents, the matrix is reduced to *P* ×*P* by removing some of the rows and columns using SVD. In order to reduce the loss of information, only the least significant part of the frequency matrix is ignored. The documents processed by the SVD technique can be used for interdocument similarity comparison, while the top *N* matching outputs are output. The retrieval effect of this method is not very obvious, while the selection for the low-dimensional space is often difficult, limiting the space for the use of this technique.

In addition, transfer learning methods are often used by means of similarity dictionaries. Similarity dictionaries are often used to deal with word ambiguity, and the technique treats a query as a concept. User input is often too homogeneous and has a lot of ambiguity, and it is better to expand the user input into multiple query words with similar meanings for joint search by query expansion methods. Therefore, the selection of extended terms can be obtained by cooccurrence with query terms. For example, the phrase finder technique represents any concept A as a tuple set, which contains all the words cooccurring with concept A and their frequency of occurrence, and the tuple set is the pseudodocument. When the user enters a query term, the system automatically calculates the relevance of the query term to the words in the pseudodocument and outputs the results in a ranked manner as query extensions for joint search. The similarity dictionary has excellent retrieval effect and high accuracy rate of query, but it is too complicated to establish the concept of association between all words in advance, and the calculation is too complicated, and the retrieval efficiency is low.

RETRACTED

The transfer learning analysis is a combination of global analysis and local analysis. Using the local feedback method to select relevant documents, the phrase finder technique in global analysis is applied to the cooccurrence idea in the selection of extension terms, which well avoids the situation that irrelevant documents may appear in local feedback and improves the query efficiency compared to the global analysis. The local clustering method in local analysis divides related documents into different clusters when selecting extensions and assumes that the most relevant extensions to the query term are all in the same cluster. However, in fact, there are often other irrelevant clusters besides the most relevant clusters that also contain some of the extension terms, and this phenomenon can be explained by topic overlap. In local clustering, the default related words are in the largest cluster, but if there is topic overlap in the largest cluster, the accuracy of the query of this method will be greatly reduced. A good query method should not have such topic overlap and must ensure that there is no significant decrease in precision for each query. The local context only selects words that cooccur with all query terms at the same time as extensions, ensuring high relevance to the maximum extent. This method was used in the INQUERY system and achieved good results on the TREC standard test set.

### 2.3. Combining Transfer Learning with Deep Neural Networks

In this paper, a graphical deep neural network modeling approach is chosen to build a sports video ontology model, in addition to combining the search term detection technique of transfer learning to build a video intelligent classification system. Firstly, the sports ontology is defined as a triple Sport Onto = (*T*, *R*, *I*), where (1) the set of nodes *O* = {Term1, Term2, Term3, ... ,Term*n*} denotes the set of terms. (2) The set of arcs belongs to (*P* ∗ *P*), which represents the binary relation on T. The relation is_a, part_of, or kind_of is satisfied between Termi and Termj. (3) O is the set of instances. The sports video ontology is modeled by Protégé according to the above definition and saved automatically as an OWL format file. The effect of modeling part of the sports video ontology is shown in Figure 3.

RETRACTED

The process of constructing ontologies through the language of transfer learning is as follows:

1. Define the goal: to describe the structure of sports video concepts, their attributes, and the relationships between them through the OWL language using ontological ideas.
2. Establish a hierarchy: Establishing a hierarchy between concepts requires that the concepts do not intersect with each other, and the subclasses of each class should be disjoint; e.g., the subclasses basketball and baseball of the ball class in the ontology of this paper do not intersect with each other. The edges in the hierarchy diagram of the ontology represent the relationship between concepts, such as Is_A, Part_of, and Kind_of.
3. Define the attributes and constraints of concepts: The hierarchy is equivalent to the skeleton of a human body, and the attributes and constraints are equivalent to the flesh and blood of a human being. There are two kinds of attributes of concepts: one describes its own information, and the other is used to represent the relationship between concepts, i.e., numerical attributes and object attributes.
4. Coding of the designed ontology using OWL language.

There are many factors that affect the similarity between concepts in ontologies, such as semantic overlap, distance similarity, literal similarity, and attribute matching. When making the similarity selection, we need to combine the ontology model structure and properties for comprehensive consideration and combine all relevant factors together for similarity calculation. After determining the similarity of concepts in the ontology, the threshold value is needed to judge the similarity between concepts. Only concepts whose similarity to the query term exceeds the threshold value are included in the query extension set during the extension term selection. There are various ways to determine the threshold value, such as artificially evaluating the similarity value between a small part of concepts in the ontology with a tentative threshold value, and if all similarities are greater than the threshold value, the tentative threshold value is reasonable. If the similarity between some concepts is less than the threshold, but the concept actually meets the system requirements, and the threshold is too large and should be reduced. Manual adjustments are made through continuous experiments until the threshold value basically meets the ontology model requirements.

RETRACTED

### 2.4. Text Detection Method Test

In this paper, the proposed methods are tested by experiments, including shot segmentation, key frame extraction, video annotation, and keyword query expansion. The video clips for validating the shot segmentation and key frame extraction methods are obtained from Tencent video, and the video clips for validating the video annotation and keyword query expansion methods are obtained from UCF101 dataset. In this paper, the proposed method and the traditional shot segmentation method with double-threshold detection are tested and compared based on the same sports video clips, and the results are shown in Figure 4. In addition, the double-threshold detection method is a computational analysis of the whole image frame to determine the video fade boundary, while the four-step method based on block matching used in this paper makes reasonable use of the feature that athletes in sports videos are usually in the center of the video, avoiding the detection of the middle block of the video and relatively saving computational time.

It can be seen from the data in the table that the efficiency of the method proposed in this paper has been improved compared with the dual-threshold detection method for lens boundary detection, which saves about 19.2%∼30.1% in time, because the dual-threshold detection algorithm is artificially set the threshold value, which is not well applicable to the sports video material selected in this paper; in addition, the dual-threshold detection method is a frame-by-frame analysis of the video to detect the mutation boundary, and the computational effort is relatively large. The automatic threshold-based histogram difference method proposed in this paper automatically sets the threshold value according to the complexity of the video content when performing shot mutation detection, and the processing of image frames takes the method of interframe statistics, which will improve computational efficiency.

## 3. Results and Analysis

### 3.1. Transfer Learning-Based Accuracy Testing

As shown in Figure 5, the evaluation results of this paper's footage segmentation method are based on the three parameters of check-all rate, check-accuracy rate, and F1. From the table, it can be seen that the method of this paper has good evaluation effect on mutation and gradient detection, in which the automatic threshold method and motion direction analysis used in this paper are well applied to the sports video material selected in this paper, which plays a decisive role in the improvement of the detection rate and accuracy rate. The retrieval of videos will make the video content richer, and video retrieval has become a key topic for researchers to study.

RETRACTED

Selecting appropriate video features can present a better video retrieval effect. In this paper, the shortcomings of existing methods are comprehensively analyzed in video retrieval, and corresponding improvement methods are proposed in lens segmentation, key frame extraction, video annotation methods, and query expansion methods. The histogram difference method based on automatic threshold, which sets its own threshold according to the complexity of image content, improves the accuracy of lens mutation detection; the key frame extraction method based on clustering and optical flow analysis, which combines clustering analysis and motion analysis while avoiding the shortcomings of each, increases the flexibility of the number of key frames extracted while reducing the computation; regarding the improvement based on the traditional deep neural network, the ontology-based keyword query expansion method analyzes and expands the semantic meaning of the user input words to be retrieved and jointly searches the expanded words with the query words to improve the accuracy of retrieval.

In order to evaluate the algorithm more accurately, two parameters, fidelity and matching degree, are chosen to evaluate the key frame extraction method in this paper. In order to clearly verify the feasibility of the key frame extraction method based on clustering and optical flow analysis proposed in this paper, the experiments in this paper compare the key frame extraction method based on clustering and the method in this paper based on some shots in video sports_3, and the results are shown in Figure 6.

This data shows that the key frame extraction method based on clustering and optical flow analysis proposed in this paper is better than the clustering-based key frame extraction method in terms of key frame extraction effect, both in terms of fidelity and matching degree. The clustering-based method clusters all image frames according to the difference degree when performing key frame extraction, which is effective for key frame extraction, but the number of clustering centers needs to be set in advance; i.e., the number of key frames is fixed.

RETRACTED

In sports video clips, the amount of important information in the footage varies due to the different degrees of description of motion information in the footage, and the traditional clustering analysis method extracts a fixed number of key frames, which usually has missed detection for sports videos with diverse motion information. The key frame extraction method based on clustering and optical flow analysis proposed in this paper combines clustering analysis with optical flow analysis and performs optical flow analysis again for video frames with relatively large amount of motion information. This method further analyzes the motion image frames, which can avoid the fixed number of extracted key frames in the clustering method and improve the fidelity and matching degree of key frame extraction.

### 3.2. Video Content Analysis

Among them, the reference key frames are voted by relevant video researchers, which can represent the video content information in theory. From the figure, we can see that the proposed method is basically similar to the reference key frames in terms of the number of extracted key frames, and from the content expression, except for the slight difference of individual video frames, the overall is similar and can well express the video content information. The clustering-based key frame extraction method is significantly less than the reference key frame in terms of the number of extracted key frames, and in terms of the content, the number of extracted key frames is relatively small, and the expression of the video content is not comprehensive, especially in the expression of motion details that is not as detailed as the method in this paper. The fundamental reason is that the method proposed in this paper performs additional optical flow analysis for video frames with more motion based on the clustering analysis of video frames, so that the extracted key frames describe the video motion information in more detail and therefore better represent the video content.

The video annotation method proposed in this paper is based on the extraction and classification of video frame features by convolutional neural network, so the effectiveness of the feature extraction method represents the effectiveness of the video annotation method. In order to achieve better validation, this paper tests the neural network and the improved network by UCF101 dataset, and the accuracy and completeness rates of this paper are shown in Figure 7. It can be seen that the improved convolutional neural network proposed in this paper performs better than the deep neural network on the same dataset, which indicates that this paper has improved the feature recognition ability of the network by modifying the parameters and structure of the deep neural network, and the results are better than those of the traditional deep neural network in both the accuracy and completeness. In addition, due to the reduction of network parameters in this paper, the convergence of the network is accelerated, and the computational efficiency of the network is significantly improved in this experiment, which is of great significance for the video retrieval.

RETRACTED

In order to better verify the effectiveness of the method in this paper, the sports ontology was chosen as the domain ontology, and 5000 sports articles and news corpus crawled online were used as the training set to construct the connectivity graph. The search completion rate, search accuracy rate, and reconciliation average are used as the evaluation criteria of the retrieval method. In this paper, we use the dataset mentioned in the previous section to compare the keyword query expansion method based on sports ontology and the word association matrix query expansion method and use the retrieved text “four people play basketball in the park” to obtain the keywords in the keyword set to be retrieved after text preprocessing “four,” “people,” “park,” “play,” and “basketball,” and the extended keywords and the corresponding similarity are obtained for these keywords based on the method proposed in this paper, as shown in Figure 8.

The input retrieved text “four people playing basketball in the park” was preprocessed, and query expanded to obtain the extended keyword set, which was sorted by similarity value from largest to smallest. The evaluation results of this retrieval method outperformed the word association matrix-based method, with the accuracy, completeness, and summation averages improving by 5.83%, 1.82%, and 6.32%, respectively, indicating that the query expansion method based on sports ontology proposed in this paper can improve the query effect and can complete the video retrieval task well.

By comparing this method with the traditional keyword-based retrieval method, different numbers of videos were selected to evaluate the two methods based on the search completion rate and the search accuracy rate. The number of videos retrieved by the traditional keyword-based video retrieval method is much higher than the number of manual retrievals, but the proportion of correct retrievals is very small, because the traditional keyword-based retrieval method uses manual annotation, and the annotation of video materials is not accurate due to the influence of too many subjective factors. The results of this paper are better than those of the keyword-based retrieval method in terms of both completeness and accuracy, indicating that the convolutional neural network structure proposed in this paper provides relatively accurate annotation of videos, and the ontology-based query term expansion method also plays a significant role in improving the retrieval results. From the data, the video retrieval method based on convolutional neural network proposed in this paper reduces the redundancy phenomenon of video retrieval to a certain extent and can basically meet the retrieval needs of users.

RETRACTED

## 4. Conclusion

The histogram difference method based on automatic threshold proposed in this paper takes a frame-by-frame statistical approach in performing shot mutation detection to reduce the computational effort to a certain extent, and the reasonable setting of threshold value by the automatic threshold method also plays a key role in the accurate segmentation of video shots. In this paper, the shortcomings of existing methods are comprehensively analyzed in video retrieval, and corresponding improvement methods are proposed in shot segmentation, key frame extraction, video annotation methods, and query expansion methods. Combined with the characteristics of sports video, this paper proposes a key frame extraction method based on clustering and optical flow analysis, and experimental comparison with the traditional clustering method. Since the traditional clustering method requires a preset number of cluster centers when performing cluster analysis, which also limits the number of key really extracted, making the method too inflexible when performing key frame extraction, the method in this paper extracts key frames by combining. By comparing this method with the traditional keyword-based retrieval method, different numbers of videos were selected to evaluate the two methods based on the search completion rate and the search accuracy rate. For the user's query words, the ontology-based keyword query expansion method proposed in this paper reasonably expands the query words based on semantics to form an extended word set, which is jointly queried with the query words, and the experimental comparison with the extended query method based on word association matrix shows that this method is higher than the word association matrix-based method in terms of reconciliation mean, which proves the effectiveness of this method. In the future, news corpus crawled online should be used as the training set to construct the connectivity graph.

## Figures and Tables

**Figure 1:** Structure of the redesigned neural network.

**Figure 2:** Transfer learning-based retrieval mechanism.

**Figure 3:** Internal structure of ontology based on transfer learning.

RETRACTED

**Figure 4:** Comparison of detection times.

**Figure 5:** Check rate, accuracy rate, and F1 test results.

**Figure 6:** Comparison of key frame extraction results between this method and clustering-based methods.

**Figure 7:** Accuracy and completeness of transfer learning methods.

**Figure 8:** Keyword-based video search results.

## Data Availability

The data used to support the findings of this study are available from the corresponding author upon request.
